The article "An Immune-Related Prognostic Risk Model in Colon Cancer by Bioinformatics Analysis" was retracted in 2023. Reasons: unreliable results or conclusions; concerns about the data; concerns about the peer review; concerns about the citations.

# An Immune-Related Prognostic Risk Model in Colon Cancer by Bioinformatics Analysis

**DOI:** 10.1155/2022/3640589

**Published:** 2022-08-27

**Authors:** Qing Lai, Haifei Feng

**Affiliations:** Department of Gastroenterology, The First People's Hospital of Xiaoshan Hangzhou, Hangzhou 311200, China

## Abstract

Colon cancer is one of the leading malignancies with poor prognosis worldwide. Immune cell infiltration has a potential prognostic value for colon cancer. This study aimed to establish an immune-related prognostic risk model for colon cancer by bioinformatics analysis. A total of 1670 differentially expressed genes (DEGs), including 177 immune-related genes, were identified from The Cancer Genome Atlas (TCGA) dataset. A prognostic risk model was constructed based on six critical immune-related genes (C-X-C motif chemokine ligand 1 (CXCL1), epiregulin (EREG), C-C motif chemokine ligand 24 (CCL24), fatty acid binding protein 4 (FABP4), tropomyosin 2 (TPM2), and semaphorin 3G (SEMA3G)). This model was validated using the microarray dataset GSE35982. In addition, Cox regression analysis showed that age and clinical stage were correlated with prognostic risk scores. Kaplan–Meier survival analysis showed that high risk scores correlated with low survival probabilities in patients with colon cancer. Downregulated TPM2, FABP4, and SEMA3G levels were positively associated with the activated mast cells, monocytes, and macrophages M2. Upregulated CXCL1 and EREG were positively correlated with macrophages M1 and activated T cells CD4 memory, respectively. Based on these results, we can conclude that the proposed prognostic risk model presents promising novel signatures for the diagnosis and prognosis prediction of colon cancer. This model may provide therapeutic benefits for the development of immunotherapy for colon cancer.

## 1. Introduction

Colon cancer is a common gastrointestinal malignant disease and the leading cause of cancer-related mortality worldwide [1]. In 2018, an estimated 106,180 new cases and 52,580 deaths of colon cancer are projected to occur in the United States [2]. A retrospective cohort study of the SEER colorectal cancer registry estimated that the incidence rate for colon cancer will increase by approximately 90% in 2030 [3]. According to statistics in 2022, the overall 5-year survival rate for patients with colon cancer is 64%, and that for patients at advance stage is 14% (https://www.cancer.net/cancer-types/colorectal-cancer/statistics). Currently, colon cancer is generally treated by colectomy and adjuvant chemotherapy; however, adjuvant therapy, especially containing oxaliplatin, has considerable toxicity and may induce peripheral neuropathy [4, 5]. Pathophysiological assessment, therapeutic decisions, and prognostic predictions for colon cancer mainly rely on factors with a cancer cell-centric focus, such as the TNM staging system and molecular markers [6, 7]. Previous studies have pointed that immune microenvironment influences the development of colon cancer [8, 9]. Therefore, immune cells may be a promising source of novel diagnostic and prognostic biomarkers for colon cancer.

The article "An Immune-Related Prognostic Risk Model in Colon Cancer by Bioinformatics Analysis" was retracted in 2023. Reasons: unreliable results or conclusions; concerns about the data; concerns about the peer review; concerns about the citations.

Many diagnostic and prognostic biomarkers of colon cancer, including genes, noncoding RNAs, and immune cells, have been identified by preclinical and clinical studies [7, 10–13]. Bioinformatics analysis and microarray techniques provide a powerful tool to explore gene regulation patterns, molecular mechanisms, and tumor progression or prognosis [13, 14]. For instance, Jung et al. [13] showed that nine of 34 selected candidate marker genes had high confidence in the diagnosis of colon cancer. Yang et al. [15] identified that 20 hub genes, including TIMP1, CXCL5, and COL1A1, had potential values in the diagnosis, prognosis, and treatment of colon cancer based on bioinformatics analysis of GSE44076.

Recent studies in tumor microenvironment showed that immune cell infiltration plays crucial roles in the progression of colon cancer [16, 17]. Evaluation of the densities of lymphocyte populations at tumor center, and tumor margin plays an essential complementary role to the tumor staging system in relapse and mortality prediction in colon cancer [18]. By assessing immune infiltration in tumor microenvironment constitutes, the response to existing immune checkpoint inhibitors can be accurately predicted, thereby developing novel immunotherapeutic strategies for colon cancer [9]. Immune cell compositions and infiltration profile have higher prognostic value in colon cancer, even higher than clinical factors [7, 19, 20]. However, the prognostic markers in immune cell infiltration profile of colon cancer remains unclear.

In this study, bioinformatics analysis was conducted to identify prognostic biomarkers related to immunity in colon cancer. Also, a recently developed computational method called the cell type identification by estimating relative subsets of RNA transcripts (CIBERSORT) was used to identify biomarkers associated with immune cell infiltration profile in colon cancer. Here, an immune-related prognostic risk model was established for colon cancer by bioinformatics analysis. This model contributes to the diagnosis and prognosis of colon cancer and the development of immunotherapy.

## 2. Materials and Methods

### 2.1. Data Collection

Gene expression profiling by the microarray dataset GSE39582 (GPL570, [HG-U133_Plus_2] Affymetrix Human Genome U133 Plus 2.0 Array) was downloaded from the Gene Expression Omnibus (GEO; https://www.ncbi.nlm.nih.gov/geo/) database. The dataset consisted of 585 samples, including 566 colon cancer samples and 19 nontumoral colorectal mucosae (control samples). The gene expression from RNA-seq of colon cancer in The Cancer Genome Atlas (TCGA), including 430 colon cancer samples and 39 adjacent nontumoral tissues, was downloaded from the UCSC Xena (https://xenabrowser.net/datapages/).

The article "An Immune-Related Prognostic Risk Model in Colon Cancer by Bioinformatics Analysis" was retracted in 2023. Reasons: unreliable results or conclusions; concerns about the data; concerns about the peer review; concerns about the citations.

### 2.2. Data Preprocessing

Data preprocessing was performed for the GSE39582 dataset using the affy package, including RNA correction and data normalization. The *R* package was used for the processing of data from TCGA. The HUGO Gene Nomenclature Committee (HGNC; https://www.genenames.org/) database was used for gene (protein_coding) annotation.

### 2.3. Identification of Differentially Expressed Genes (DEGs)

DEGs in colon cancer were identified from the TCGA data. Data were addressed using the Limma package (version 3.34.0; https://bioconductor.org/packages/release/bioc/html/limma.html), with the criteria of adjusted *p* value < 0.05 and |log2FC (fold-change)| ≥ 1. Also, the hierarchical clustering of DEGs was carried out using the pheatmap (version 1.0.8; https://cran.r-project.org/package=pheatmap). Immune-related genes were identified from the Immunology Database and Analysis Portal (ImmPort). The common genes of DEGs and immune-related genes in the ImmPort database were used for further analysis.

### 2.4. Enrichment Analysis

Gene ontology (GO) categories, including biological process, cellular component, and molecular functions, and Kyoto Encyclopedia of Genes and Genomes (KEGG) pathways significantly associated with DEGs were collected. The Metascape tool was used for the enrichment analysis of KEGG pathways. The GO terms were retrieved from the DAVID database (version 6.8; https://david.ncifcrf.gov/). Criteria for the significant items were minimum count ≥3, enrichment factor <1.5, and *p* < 0.05. Functional enrichment analysis was visualized using the ggplot2 in *R* (https://ggplot2.org). Gene set enrichment analysis (GSEA) was performed for immune-related DEGs using the clusterProfiler package [21].

### 2.5. Construction of the Protein-Protein Interaction (PPI) Network

PPI interactions across DEGs were extracted from the STRING database (version 11.0; https://string-db.org/cgi/input.pl). The PPI network for immune-related DEGs was established using Cytoscape (version 3.8.0; https://apps.cytoscape.org/apps/all). Core modules from the PPI network were determined using the MCODE plugin in Cytoscape (https://apps.cytoscape.org/search?q=MCODE). Significant modules were selected using the threshold of score ≥10.0 (density).

The article "An Immune-Related Prognostic Risk Model in Colon Cancer by Bioinformatics Analysis" was retracted in 2023. Reasons: unreliable results or conclusions; concerns about the data; concerns about the peer review; concerns about the citations.

### 2.6. Identification of Prognosis-Related Genes

Cox regression analysis of the multistep AIC (stepAIC) algorithm [22] was used to screen the prognosis-related DEGs. Significant items were identified when *p* < 0.05. Then, a prognostic model was constructed for risk assessment, and the risk score of each sample in the TCGA and GSE39582 datasets was calculated. The cutoff values of each prognosis-related DEG in both TCGA and GSE39582 datasets were identified, and samples in both the datasets were allocated to high- and low-risk groups accordingly. The *R* survival [23] and survminer [24] packages were used for the survival analysis using the Kaplan–Meier (KM) method. The pROC package [25] was used to construct the receiver operating characteristic (ROC) curves of prognosis-related DEGs.

### 2.7. Correlation Analysis of Clinical Factors and Prognostic Risk Score

Clinical factors associated with the prognostic risk score based on the TCGA dataset were identified using Cox regression analyses. The forestplot package in *R* was applied to construct the forest plot of clinical factors.

### 2.8. Immune Cell Infiltration Analysis of Prognostic Genes

Correlation of prognostic genes with immune cell infiltration was analyzed using the CIBERSORT algorithm [26]. Immune cell infiltration matrix was constructed using the gene expression profiling in TCGA and profiling tumor-infiltrating immune cells (*n* = 22) by CIBERSORT. Results were visualized using the ggplot2 (box plot) and the pheatmap (heatmap) packages.

## 3. Results

### 3.1. DEGs Identification

Using the TCGA dataset, a total of 1670 DEGs were identified, including 763 upregulated and 907 downregulated DEGs (Figures 1(a) and 1(b)). Also, 2483 immune-related genes were identified from the ImmPort database, including 177 DEGs (Table S1).

### 3.2. Functional Enrichment Analysis

Functional enrichment analysis was conducted for all DEGs. Results exhibited that DEGs were associated with GO biological processes, including “cell chemotaxis,” “cytokine-mediated signaling pathway,” “cellular response to chemokine,” and “leukocyte migration” with the molecular functions of “receptor-ligand activity,” “growth factor activity,” and “cytokine receptor binding” (Figure 2(a)). Also, these genes were associated with multiple KEGG pathways, including “cytokine-cytokine receptor interaction,” “chemokine signaling pathway,” “IL-17 signaling pathway,” “TNF signaling pathway,” “NF-kappa B signaling pathway,” and “toll-like receptor (TLR) signaling pathway” (Figure 2(b)).

GSEA analysis presented that the immune-related DEGs were associated with 1026 GO biological processes, including “multicellular organismal homeostasis,” “positive regulation of MAPK cascade,” and “regulation of hormone levels” (Figure 3(a)), and 89 KEGG pathways, including “MAPK signaling pathway,” “calcium signaling pathway,” “neuroactive ligand-receptor interaction,” “GnRH signaling pathway,” and “gap junction” (Figure 3(b)). The GSEA plot showing the top five biological process terms and KEGG pathways associated with DEGs are shown in Figures 3(c) and 3(d), respectively.

The article "An Immune-Related Prognostic Risk Model in Colon Cancer by Bioinformatics Analysis" was retracted in 2023. Reasons: unreliable results or conclusions; concerns about the data; concerns about the peer review; concerns about the citations.

### 3.3. PPI Network of Immune-Related DEGs

The PPI network was constructed for 177 immune-related DEGs, consisting of 908 interaction pairs (edges) and 167 nodes (DEGs; Figure 4(a)). One module with a score of 18.762, 22 nodes, and 197 edges was identified in the PPI network (Figure 4(b)). Top 22 nodes with top high interaction degrees in the PPI network were included in the module, including CXCL12, CXCL2, CXCL5, CXCL11, and CXCL10.

### 3.4. Identification of Prognosis-Related DEGs

Prognosis-related DEGs were selected using the stepAIC algorithm from 177 immune-related DEGs. Finally, six immune-related DEGs, including CXCL1 (upregulated), FABP4 (downregulated), EREG (upregulated), CCL24 (eotaxin-2; upregulated), TPM2 (downregulated), and SEMA3G (downregulated), were identified as the prognosis-related DEGs and were used to construct a prognostic risk assessment model. Samples in both TCGA and GSE39582 datasets were divided into the high- and low-risk groups according to the prognostic risk assessment model. KM survival analysis showed significant differences in the survival probabilities between patients of high- and low-risk groups in TCGA (*p*=0.00065, Figure 5(a)) and GSE39582 (*p*=0.047, Figure 5(b)). Patients with high-risk scores had low survival probabilities compared with patients with low-risk scores. In addition, ROC curves of six prognosis-related DEGs indicated that CXCL1 and FABP4 had high accuracies in predicting survival in colon cancer patients (AUC >0.9; Figures 5(c) and 5(d)).

### 3.5. Correlation between Clinical Factors and Prognostic Risk Score

Eight clinical factors, including age, gender, race, stage, pathologic *M*, pathologic N, pathologic *T*, and prior malignancy, were extracted from TCGA data and used for Cox regression analyses. Univariate Cox regression analysis presented that age, stages III and IV, pathologic *M*, pathologic N, and pathologic *T*4 were significantly associated with the prognosis (*p* < 0.05; Figure 6(a)). Further multivariate Cox regression analysis displayed that age and stage IV were correlated with the prognostic risk scores of patients with colon cancer (*p* < 0.05; Figure 6(b)). Also, high risk scores correlated with low survival probabilities in colon cancer patients, irrespective of age (Figures 7(a) and 7(b)) and stage (Figures 7(c) and 7(d)).

The article "An Immune-Related Prognostic Risk Model in Colon Cancer by Bioinformatics Analysis" was retracted in 2023. Reasons: unreliable results or conclusions; concerns about the data; concerns about the peer review; concerns about the citations.

Using the CIBERSORT algorithm, we found that the downregulated genes TPM2, FABP4, and SEMA3G were positively related to the activated mast cells, monocytes, and macrophages M2 (Figure 8). Upregulated genes CXCL1 and EREG were positively associated with macrophages *M*1 and activated *T* cells CD4 memory, respectively. Also, patients with colon cancer had higher percentages of activated *T* cells CD4 memory, *T* cells follicular helper, macrophages *M*0 and *M*1, resting/activated dendritic cells, and neutrophils, and lower percentages of B cells naïve, plasma cells, *T* cells CD4 memory resting, activated NK cells, monocytes, macrophages *M*2, and activated mast cells compared with healthy controls (*p* < 0.01; Figure S1).

## 4. Discussion

A prognostic risk assessment model was constructed for colon cancer using the expression signature of six immune-related DEGs, including CXCL1 (upregulated), EREG (upregulated), CCL24 (eotaxin-2; upregulated), FABP4 (downregulated), TPM2 (downregulated), and SEMA3G (downregulated). CXCL1 and FABP4 genes had higher accuracies in predicting the prognosis in colon cancer in TCGA and GSE35982 datasets compared with other four genes. In addition, TPM2, FABP4, and SEMA3G genes were positively correlated with activated mast cells, monocytes, and macrophages *M*2. However, CXCL1 and EREG genes were positively associated with macrophages *M*1 and activated *T* cells CD4 memory, respectively. These results showed that these biomarkers were involved in the prognosis of patients with colon cancer by regulating the immune microenvironment.

In this study, six genes (CXCL1, EREG, CCL24 (eotaxin-2), FABP4, TPM2, and SEMA3G) were selected to establish a prognostic risk assessment model for colon cancer. Among them, TPM2 and tropomyosin 2*β* was decreased in the colon cancer tissue compared with normal tissues [27, 28]. Xiao et al. showed that TPM2 is associated with motility and the cytoskeleton, which may regulate tumor cell invasion and migration [29]. CXCL1 was originally cloned from fibroblast [30]. Cao et al. found that CXCL1 expression was significantly increased in hepatocellular carcinoma tissues compared to normal tissues. The high CXCL1 expression could promote proliferation and invasion of hepatocellular carcinoma cells through the NF-ĸB-dependent pathway, with poorer overall survival compared to low expression [31]. Also, CXCL1-mediated cancer growth and progression is mediated by neutrophil recruitment [32, 33]. Besides, FABP4 was an independent risk factor in colon cancer (100 patients and 100 controls; odds ratio = 1.916, 95% CI 1.340–2.492) [34]. The prognostic risk model of six immune-related DEGs presented the potential prognostic value in colon cancer clinically.

The article "An Immune-Related Prognostic Risk Model in Colon Cancer by Bioinformatics Analysis" was retracted in 2023. Reasons: unreliable results or conclusions; concerns about the data; concerns about the peer review; concerns about the citations.

Immune cell infiltration plays crucial roles in the pathogenesis, progression, prognosis, and treatment of tumors and other diseases [16, 17, 35, 36]. The composition or infiltration profile of immune cells has a high prognostic value in colon cancer, even higher than clinical factors [7, 19, 20]. Tumor progression is enhanced by M2 polarization of macrophages, recruitment of neutrophils, dendritic cells, T cells, NK cells, and CD14^+^ monocytes, by promoting the immunosuppressive environment [37–40]. Jackute et al. showed that tumor-infiltrating *M*2 and *M*1 macrophages were both related to overall survival of non-small-cell lung cancer (NSCLC) [41]. High infiltration of *M*1 and *M*2 macrophages was associated with increased and reduced overall survival in NSCLC (*p* < 0.05), respectively. Lan et al. showed that M2 macrophages induce colon cancer cell migration and invasion [42, 43]; however, *M*1 macrophages present the opposite effect [44]. Also, *M*2 macrophage-conditioned medium can induce colorectal adenocarcinoma cell migration by enhancing CD47 expression [45]. Our present study exhibited that the expression of downregulated FABP4, TPM2, and SEMA3G genes was positively correlated with the composition of *M*2 macrophages, and upregulated CXCL1, EREG, and CCL24 (eotaxin-2) were negatively correlated with *M*2 macrophages. Also, lower macrophages *M*2 was found in colon cancer tumor tissues compared with control tissues. These results showed that the six gene signatures play crucial roles in the pathogenesis, progression, and prognosis of colon cancer through tumor infiltration of *M*2 macrophages.

Furthermore, downregulated FABP4, TPM2, and SEMA3G genes were positively associated with the infiltration of activated NK and mast cells, and monocytes, but were negatively related to neutrophils, *M*1 macrophages, and *T* cells. Upregulated CXCL1 gene was positively correlated with *M*1 macrophages and neutrophils, while upregulated EREG and CCL24 (eotaxin-2) were correlated with eosinophils. Eosinophils and neutrophils are antitumoral effector immune cells. Increased infiltrating eosinophils in colon cancer tissues are associated with a better prognosis [46]. Neutrophil infiltration has been reported to be a favorable prognostic factor in early stage (I and II) of colon cancer [47]. Neutrophils promote resistance to radiotherapy in cervical cancer [48]. Also, tumor-associated neutrophils mediate immunosuppression in breast cancer [49]. These results showed that these genes were involved in the progression and prognosis of colon cancer by regulating immunosuppression and tumor microenvironment. Based on results mentioned above, this immune-related prognostic model established in this study can serve as a robust prognostic biomarker for colon cancer and provide therapeutic benefits for the development of novel immunotherapy.

The article "An Immune-Related Prognostic Risk Model in Colon Cancer by Bioinformatics Analysis" was retracted in 2023. Reasons: unreliable results or conclusions; concerns about the data; concerns about the peer review; concerns about the citations.

## 5. Conclusions

In this study, by bioinformatics analysis, six immune-related genes (CXCL1, EREG, CCL24, FABP4, TPM2, and SEMA3G) were found to be significantly associated with the prognosis of colon cancer. Based on these six genes, an immune-related prognosis model was constructed for colon cancer. This prognostic model presented significant correlation with the infiltration of immune cells, proving its critical role in the tumor immune microenvironment. Current study contributes to the understanding of immune-related genes in colon cancer and provides novel potential diagnostic and prognostic biomarkers. Further, *in vitro* and *in vivo* studies are needed to be performed to validate this prognostic model and immune-related biomarkers.

## Figures and Tables

**Figure 1:** The profile of differentially expressed genes (DEGs). (a) The volcano plot of DEGs. (b) The hierarchical clustering of DEGs.

**Figure 2:** Functional enrichment analysis of differentially expressed genes (DEGs). (a, b) Gene Ontology terms and KEGG pathways associated with DEGs, respectively.

**Figure 3:** Gene set enrichment analysis (GSEA) of differentially expressed genes (DEGs). (a, b) The ridgeline plots of top 10 biological processes and KEGG pathways associated with DEGs in colon cancer, respectively. (c, d) The GSEA plots of the top five biological processes and KEGG pathways associated with DEGs, respectively.

**Figure 4:** Protein-protein interaction (PPI) network of immune-related genes in colon cancer. (a) The PPI network based on 177 differentially expressed immune-related genes (immune-related DEGs). (b) The significant module (top 22) in the PPI network. Color depth and node size correspond to interaction degree. Orange and blue colors denote low and high degree, respectively.

**Figure 5:** Survival analysis of the prognostic risk assessment model in colon cancer. (a, b) Kaplan–Meier (KM) survival analysis in the TCGA and GSE39582 dataset. (c, d) Receiver operating characteristic (ROC) curves of six genes in TCGA and GSE39582 dataset. AUC, area under ROC.

**Figure 6:** Correlation analysis of clinical factors with a prognostic risk score of colon cancer in the TCGA database. (a, b) univariate and multivariate Cox regression analysis of clinical factors associated with the prognostic risk score in TCGA dataset, respectively. HR, hazard ratio; CI, confidence interval.

The article "An Immune-Related Prognostic Risk Model in Colon Cancer by Bioinformatics Analysis" was retracted in 2023. Reasons: unreliable results or conclusions; concerns about the data; concerns about the peer review; concerns about the citations.

**Figure 7:** Survival analysis of patients with colon cancer based on different age and stage groups based on TCGA database. (a, b) Kaplan–Meier (KM) survival curves of patients with age ≤68 and >68 groups. (c, d) Kaplan–Meier (KM) survival curves of TCGA patients at different stage groups. Patients were divided into high- and low-risk groups based on the prognostic risk assessment model. Immune cell infiltration in patients with colon cancer.

**Figure 8:** Immune cell infiltration in colon cancer based on prognostic-related genes. Blue and red colors denote negative and positive correlation, respectively.

## Data Availability

The data used to support the findings of this study are available from the corresponding author upon request.

## Supplementary Materials

Supplementary Materials Table S1: the 177 immune-related genes that differentially expressed between colon cancer tissues and adjacent nontumoral tissues based on The Cancer Genome Atlas (TCGA) database. Figure S1: cell composition of 22 immune cells in colon cancer patients. The symbols ^*∗*^, ^*∗∗*^, ^*∗∗∗*^, and ^*∗∗∗∗*^ represent *p* < 0.05, 0.01, 0.001, and 0.0001, respectively.
